The article "Interactive Model of Rural Tourism and New Socialist Countryside Construction Using Deep Learning Technology" was retracted in 2023. Reasons: signs of a paper mill; suspected computer-generated content; unreliable results or conclusions; concerns about the data.

# Interactive Model of Rural Tourism and New Socialist Countryside Construction Using Deep Learning Technology

**DOI:** 10.1155/2022/2620548

**Published:** 2022-07-05

**Authors:** Yupeng Chen

**Affiliations:** School of International Education, Yiwu Industrial and Commercial College, Yiwu 322000, China

## Abstract

China has proposed two major measures to address the “three rural issues”: the first is to abolish the agricultural tax, which has been in place for over 2000 years; the second is to propose the construction of a new socialist countryside, which would mark the end of the old era and the beginning of the new. As a result, this paper employs in-depth learning technology to enhance rural tourism development and the creation of a new socialist countryside. This paper investigates deep-learning-based rural tourism and the creation of a new socialist countryside. Because MSE and MAE reflect the prediction error score, the lower the value, the better the recommendation accuracy. The MSE value of the machine learning algorithm is 2.456, the MSE value of the data mining algorithm is 2.324, and the MSE value of the convolution neural network algorithm is 2.102, when the number reaches 80. It can be concluded that the convolution neural network algorithm proposed in this paper has the lowest MSE and MAE values of the three methods, implying that the convolution neural network algorithm is the best of the three. The use of the convolution neural network algorithm to implement the scientific concept of development and the construction of a new socialist countryside is an important part of creating a harmonious society that fully meets the central government's objectives and requirements for the construction of a new socialist countryside.

## 1. Introduction

The National Tourism Administration has opened up a new field of tourism development, providing a new path for developing rural tourism resources, adjusting agricultural industrial structure, expanding employment, and promoting farmers' income and wealth, as well as being an important measure to promote the development of new socialist countryside. China has proposed two major measures to address the “three rural issues”: the first is to abolish the agricultural tax, which has been in place for over 2000 years, and the second is to construct a new socialist countryside. This signals the end of an era and the start of a new one. The logic behind it is to move away from urban-rural division and toward urban-rural integration, which is the process of integrating the city and the countryside into an organic whole [1, 2]. In this context, some rural areas with abundant natural or humanistic tourism resources have achieved remarkable results by promoting new rural construction through rural tourism, which not only opens up a new field of tourism development, but also serves as an important tool for promoting new socialist rural construction [3]. Building a new socialist countryside is a critical strategic task for adapting to the “three rural issues,” realising the goal of a prosperous society, and establishing a harmonious socialist society. Its realistic foundation is the widening divide between urban and rural areas, as well as the difficulty for the vast rural population to share the benefits of modernization fairly. We must fully develop and utilise agricultural resources, adjust and optimise rural industrial structure, improve rural civilization and farmer quality, promote the construction of a civilised rural style, and mobilise farmers' enthusiasm and creativity for production [4, 5].

The article "Interactive Model of Rural Tourism and New Socialist Countryside Construction Using Deep Learning Technology" was retracted in 2023. Reasons: signs of a paper mill; suspected computer-generated content; unreliable results or conclusions; concerns about the data.

The difference between deep learning [6, 7] and machine learning [8–10]: traditional machine learning mainly relies on manual definition of features, while deep learning algorithm can learn features independently, and represents the learned deep feature relationship between users and objects in the same space. Convolutional neural network (CNN) is a kind of deep neural network in deep learning. It is a shared weight architecture based on convolution kernel, and the feature convolution neural network used to scan the hidden layer is mainly used to identify the image data that is translated, scaled, and distorted to some extent. Because the general CNN structure is mostly an end-to-end system, it can implicitly learn the features related to the task directly from the data, without too much human intervention, and without a lot of expert domain knowledge. The function of convolution layer is to convolve the input layer and transfer the result to the next layer. Convolution operation can be seen as a process in which one function performs linear transformation on another function and maps it to a new value.

This paper builds an interactive model between rural tourism and the construction of a new socialist countryside based on the convolution neural network algorithm under deep learning. Training data is used to build the interactive model. It can directly predict the probability value of tourism classification that tourists are interested in when the characteristic attributes of new tourists are obtained [11, 12]. Different characteristic layers of new socialist rural construction are obtained using the convolution kernel sliding on the characteristic matrix of rural tourism. By combining the outputs of neurons in one layer, the pooling layer reduces the amount of data calculations. Maximum and average pooling are the most common pooling types. Pooling is used to create a smaller characteristic matrix, which is then linked to the next layer. The convolution neural network algorithm is an important part of building a harmonious society and fully conforms to the central government's objectives and requirements for building a new socialist countryside [13]. It is an important measure to implement the scientific concept of development and build a new socialist countryside under the convolution neural network algorithm.

The article "Interactive Model of Rural Tourism and New Socialist Countryside Construction Using Deep Learning Technology" was retracted in 2023. Reasons: signs of a paper mill; suspected computer-generated content; unreliable results or conclusions; concerns about the data.

In this paper, I mainly put forward the following innovative contents:

1. in this paper, a CNN model is constructed. CNN model is one of forward neural network models. In order to better understand it, we first introduce the connection mode and optimization method of forward neural network structure, and then introduce the characteristics of CNN. A typical CNN can be found from the figure that it is mainly composed of five parts, namely, input layer, convolution layer, pooling layer, full connection layer, and output layer.
2. The experiment on the influence of parameter setting on the model shows that the sensitivity and accuracy of the convolution neural network algorithm proposed in this paper are the first among the three algorithms. Compared with other algorithms, CNN algorithm can make good use of some basic information and comment text information, and also make use of the hidden interaction between these information, which other algorithms do not have. Therefore, their accuracy and sensitivity are lower than those of convolution neural network algorithm.

The first chapter introduces the background and significance of rural tourism and the construction of new socialist countryside, and then introduces the main work of this paper. The second chapter mainly introduces the relevant literature of rural tourism and the construction of a new socialist countryside. The third chapter describes the related content of deep learning technology, and puts forward a variety of models. In the fourth chapter, the experiment procedure and the results are analyzed and discussed. The fifth chapter is a summary of the full text.

## 2. Literature Review

The details were collected by making full use of the superiority of modern network, collecting the research results of rural tourism and new rural construction, reading a large number of relevant yearbooks and planning texts for analysis, induction, and summary, determining the research content, and seeking the theoretical guidance of the interactive development of rural tourism and new rural construction. The details are as follows:

Chui et al. proposed that rural tourism will become a supporting industry for building a new socialist countryside. Under the new situation, the tourism industry should take advantage of the vast space of the new socialist countryside, give full play to its own advantages, focus on the work center of “agriculture, rural areas, and farmers,” and be close to agriculture, rural areas, and farmers, so as to continuously infiltrate the tourism industry into rural areas by developing rural tourism [14]. Kim pointed out that with the transition from a traditional country to a modern country, the political opposition between urban and rural areas began to be eliminated. The most prominent thing is that farmers, like urban citizens, have obtained an abstract and equal national qualification and national rights [15]. Akinosho et al. put forward that the development of tourism economy is closely linked with the humanities and natural ecological environment. Any tourism activity is a process of material and energy exchange between human beings and the surrounding environment. Without a good ecological environment, there would be no tourism, which is especially important for the development of rural tourism [16]. Hu puts forward that rural tourism refers to a new tourism business activity that provides sightseeing, leisure, vacation, experience, entertainment, and fitness for urban people through scientific planning, development, and design in rural areas, using rural natural environment, pastoral landscape, rural animal husbandry and fishery production, farming culture, folk culture, ancient towns and villages, and pleasant life [17]. Lee et al. put forward that rural tourism can really show its significance only when it has made efforts and achieved results in protecting rural ecological environment, protecting cultural landscape and protecting ethnic customs, increasing enough employment opportunities, and driving local social and economic development at the same time [18]. Jaturapitpornchai et al. put forward that the essence of rural tourism economic development is to use the beautiful natural environment and rich national culture to attract tourists and meet their growing tourism needs [19]. Yang and Gong put forward that the rise and development of rural tourism are closely related to social and economic development. From the perspective of development history, rural tourism is under the condition of high industrialization and urbanization. Due to the increase of urban residents' income, changes in lifestyle and consumption structure, the urban residents are no longer satisfied with the living environment and tourist attractions in the city, but hopes to get out of the city, into the countryside, return to nature, and get close to nature [20]. Shen et al. put forward that in the current market economy environment, the mutual promotion of tourism, and agricultural development has been highly valued by the relevant government departments, and the function of tourism has been given a new position, which has been entrusted with the arduous historical mission of promoting the implementation of the policy of agriculture, rural areas, and farmers through tourism. This is not only an important attempt to promote the rural economy through tourism development, but also opens up a broader space for the sustainable development of tourism [21]. Liu and Liu proposed that the development of rural tourism should be based on large agricultural resources and the existing rural natural and cultural landscape in the region, and the comprehensive and diversified development of rural tourism products should be carried out. Liu and Liu also proposed to extend the rural industrial chain, attach importance to the development of agricultural product processing industry, establish enterprises with local agricultural product processing as the leader, introduce advanced planting and processing technologies, and speed up the development and production of agricultural products [22]. Miao et al. put forward that rural tourists are consumers of new rural facilities and rural tourism resources, and the success of new rural construction and rural tourism development will greatly affect the satisfaction of tourists and the reputation of destinations. Therefore, strengthening the cooperation and communication among rural residents, grass-roots governments, enterprises and institutions, tourists and other relevant stakeholders, taking into account and coordinating the interests of all parties, is an important condition for the benign interaction between new rural construction and rural tourism [23].

The article "Interactive Model of Rural Tourism and New Socialist Countryside Construction Using Deep Learning Technology" was retracted in 2023. Reasons: signs of a paper mill; suspected computer-generated content; unreliable results or conclusions; concerns about the data.

The goal of this study is to serve as a practical guide for the development of rural tourism and new rural construction in general. As a result, this paper investigates rural tourism and the construction of new socialist countryside using in-depth learning, proposes a convolution neural network algorithm, and builds an interactive model between rural tourism and the construction of new socialist countryside. Rural tourism development in the surrounding radiation areas of large- and medium-sized cities can achieve the development mode of urban spontaneous support for rural areas through market economy adjustments. The CPC's long-term improvement of its ruling philosophy resulted in the creation of a new socialist countryside using a convolution neural network algorithm. Promoting the party's overall development in rural areas in accordance with China's national circumstances is a major historical task. We should create a harmonious socialist countryside using the convolution neural network algorithm, recognise the close relationship between tourism and agriculture, and use tourism as a new way to diversify agricultural resource management without compromising agricultural development. The tourism industry, which uses a convolution neural network algorithm, can not only help nearby farmers become wealthy, but it can also attract farmers from far away to participate in tourism transportation, planting and breeding, and commodity production. Tourism not only provides farmers with a long-term source of income, but it also has a very low chance of returning them to poverty.

## 3. Deep Learning Technology

### 3.1. Basic Principle and Model of CNN

CNN is a multi-layer perceptron network model for dealing with gridded data, such as image data. The most significant difference between it and a conventional multi-layer perceptron is that CNN can reduce the number of neurons in its model by using a pooling layer [24]. The benefit of this network is that it can extract local and global features using relevant convolution operations, avoiding the time-consuming process of feature extraction and data reconstruction required by traditional recognition algorithms. It has strong representation learning capabilities, can perform both supervised and unsupervised learning, and effectively improves data accuracy and scientificity. It is possible to share CNN weights. The parameters can be reduced significantly, the network's complexity is reduced, and the network's generalisation ability is improved in this way. Translation invariance is also a feature of it. Furthermore, and perhaps most importantly, it can operate directly on images without the need for complex operations like data pre-processing and feature extraction, which is the most significant difference from traditional image processing methods [25]. A feedforward neural network is a type of CNN. To help you understand it better, well go over the feedforward neural network structure's connection mode and optimization method first and then the CNN's characteristics. The input layer, convolution layer, pooling layer, full connection layer, and output layer are the five main components of a typical CNN, as shown in the diagram. Input layer, convolution layer, pooling layer, full connection layer, and output layer are the layers that make up this system. The convolution neural network model is shown in Figure 1.

Convolution layer: the core of feature extraction of CNN is convolution layer and pool layer. Each layer of convolution layer is composed of a feature map containing multiple neurons, and the features of input data are extracted by convolution operation of convolution kernel. The calculation formula of convolution layer is as follows:

(1) $$\begin{array}{c} x_{j}^{l}=\sigma \left(\sum_{i\in h_{j}}x_{i}^{l-1}\right), \end{array}$$

where, *x*_*j*_^*l*^ represents the output eigenvalue, *σ* is the activation function, *h*_*j*_ is the convolution filter window size, and *x*_*i*_^*l*−1^ is the input eigenvalue of the previous layer.

The article "Interactive Model of Rural Tourism and New Socialist Countryside Construction Using Deep Learning Technology" was retracted in 2023. Reasons: signs of a paper mill; suspected computer-generated content; unreliable results or conclusions; concerns about the data.

Pool layer: each convolution layer is connected with a pool layer, and the output of the convolution layer is used as the input of the pool layer. The pool layer mainly extracts local information through multiple nonlinear functions, and the extraction methods are average pool and maximum pool. The calculation formula of pool is as follows:

(2) $$\begin{array}{c} x_{j}^{l}=\sigma \left(\text{pool}\left(x_{j}^{l-1}\right)\right), \end{array}$$

where, *x*_*j*_^*l*^ represents the output eigenvalue, *σ* is the activation function, pool is the pool function, and *x*_*j*_^*l*−1^ is the input eigenvalue of the previous convolution layer.

Full connection layer: after the pool layer, the full connection layer weights the features extracted from the convolution layer and the pool layer, and then classifies or predicts different tasks. The formula of the whole connection layer is as follows:

(3) $$\begin{array}{c} x^{l}=\sigma \left(K^{l}x^{l-1}\right), \end{array}$$

where, *x*^*l*^ represents the output eigenvalue, *σ* is the activation function, *K*^*l*^ is the weight value, and *x*^*l*−1^ is the input eigenvalue of the previous pool layer.

If the number of neurons in the first hidden layer of the designed feedforward neural network is the same as that of the input, then, the number of adjustable parameters is 10. If the network depth continues to increase, the training network will be slow and the satisfactory results will not be achieved [26]. Therefore, in order to directly process image data, it is necessary to reduce adjustable parameters and speed up convergence. CNN has the advantage that it can reduce the adjustable parameters of the network and speed up the training speed of the network.

### 3.2. Common Deep Learning Models

#### 3.2.1. Autoencoder

The self-encoder is composed of input layer *x*, hidden layer *h*, and output layer *y*. It is a network model with a three-layer neural network structure: the number of neurons in the input layer and output layer are the same, and the structure is shown in Figure 2 below.

Input *x* will get output *y* through the self-encoder. At this time, there will be an error between input *x* and output *y*. This error is also called reconstruction table error. Reconstruction table error can usually be defined as mean square error and cross entropy. Generally speaking, it will take different definitions according to different data [27]. The self-encoder can be used in scoring prediction, image recommendation, text recommendation, and other scenarios. In the recommendation system, the self-encoder is mainly used to learn the implicit feature representation of users and projects. It learns the implicit expression of users and projects by reconstructing the relevant information of users and projects, and then, predicts the good behavior of users through this expression [28].

The article "Interactive Model of Rural Tourism and New Socialist Countryside Construction Using Deep Learning Technology" was retracted in 2023. Reasons: signs of a paper mill; suspected computer-generated content; unreliable results or conclusions; concerns about the data.

#### 3.2.2. Cyclic Neural Network

The traditional feedforward neural network structure is ineffective at modelling sequence data, whereas the cyclic neural network is very good at it. Machine translation, speech recognition, and other fields use recurrent neural networks extensively. The cyclic structure within the recurrent neural network is what allows it to process sequence information. The current hidden layer's state, as well as the hidden layer of the next layer, is determined by the state of the input layer and the previous hidden layer at the same time, forming a cyclic neural network. The most significant difference between a cyclic neural network and a traditional neural network is that each neuron node in the hidden layer is connected as well. As a result, the output of the previous hidden layer is calculated as the input of this moment, implying that the recurrent neural network can remember information. The following formula changes the loop's hidden status.

(4) $$\begin{array}{c} s_{t}=\sigma \left(s_{t-1},x_{t}\right). \end{array}$$

The activation functions of *σ* hidden layer nodes, such as tanh function and sigmoid function, are shown in formula.

(5) $$\begin{array}{c} \tanh\left(x\right)=\frac{e^{x}-e^{-x}}{e^{x}}, \end{array}$$

(6) $$\begin{array}{c} \text{sigmoid}\left(x\right)=\frac{1}{1+e^{-x}}. \end{array}$$

The hidden state of the recurrent neural network is updated by the following formula:

(7) $$\begin{array}{c} s_{t}=g\left({\text{Wx}}_{t}+{\text{Us}}_{t-1}\right), \end{array}$$

where, *g* is a nonlinear activation function, *W* and *U* are weight matrices.

Because of the gate structure, there will be no gradient disappearance or gradient explosion when dealing with time series problems with excessive length.

(8) $$\begin{array}{c} i_{t}=\sigma W_{i}x_{t}, \end{array}$$

(9) $$\begin{array}{c} O_{t}=\sigma W_{o}x_{t}, \end{array}$$

(10) $$\begin{array}{c} f_{t}=\sigma W_{f}x_{t}. \end{array}$$

The input transformation formula is as follows:

(11) $$\begin{array}{c} \tilde{C_{t}}=\tanh\;W_{C}x_{t}. \end{array}$$

The updated formula is as follows:

(12) $$\begin{array}{c} C_{t}=f_{t}*C_{t-1} \end{array}$$

Long-term and short-term memory networks can control when to let the input enter neurons, when to remember what was learned in the previous time series, and when to let the output pass to the next timestamp. This model is powerful and has achieved milestone results in many tasks such as translation, speech recognition, and recommendation system. These operations can help improve the effectiveness of implicit expression of users and projects. At present, the recurrent neural network is mainly used in image recommendation, text recommendation, location-based social network, and point of interest recommendation.

The article "Interactive Model of Rural Tourism and New Socialist Countryside Construction Using Deep Learning Technology" was retracted in 2023. Reasons: signs of a paper mill; suspected computer-generated content; unreliable results or conclusions; concerns about the data.

### 3.3. The Key to the Development of Rural Tourism

Culture is always the most active factor in the development of tourism. Modern tourism no longer only stays on the surface of natural landscape, but also needs the enrichment of cultural elements. The ancient and profound rural culture has accumulated the essence of 5000 years of Chinese culture. Over the past thousands of years, the history has been scouring to form village dwellings with different styles. It carries rich cultural and folk information and inherits the traditional Chinese farming culture. At present, the development of rural tourism is lack of planning, and the development of rural tourism economy is mainly restricted by the lagging rural tourism infrastructure and the low quality of farmers in tourism management. The practice of developing rural tourism has proved that solving these problems must rely on the strong support of the government and strengthen the leading role of the government. China's rural areas are vast, diverse, and less affected by urbanization. The vast majority of places maintain natural features. In addition, many different styles of local customs and folk customs make rural tourism unique in the object of activities. In the face of traditional rural culture, Chinese urban culture presents another cultural form. In the process of development, Chinese urban culture has been impacted by Western culture, which has penetrated the factors of Western culture. It is a hybrid of Chinese and Western culture, and it is difficult to preserve the most original cultural face of China itself. The characteristics of “ancient, original, true, and native” formed in specific regions have unparalleled advantages of being close to nature in cities and towns and provide services for tourists to return to nature. Rural tourism planning should be coordinated with the overall regional tourism planning and urban development planning, obey, and serve the overall regional tourism planning and urban development planning, and put an end to the repeated construction and arbitrary destruction of the ecological environment.

The article "Interactive Model of Rural Tourism and New Socialist Countryside Construction Using Deep Learning Technology" was retracted in 2023. Reasons: signs of a paper mill; suspected computer-generated content; unreliable results or conclusions; concerns about the data.

Natural features, labour forms, and traditional customs are the primary sources of rural tourism resources. Natural events such as water, soil, light, and heat have a significant impact on agricultural production at all stages. As a result, there is a clear seasonality to rural tourism. We should properly handle the connection between the new rural planning and the tourism planning as we prepare the coordinated development planning for the two. We should not only make the indicators of new construction truly reflect the indicators of new construction, but also make it have the functions of tourism services, and effectively prevent random development and construction, that is, the overall construction of the new countryside should take into account the development needs of rural tourism, provide support for rural tourism development, and serve the construction of the new countryside at the same time as rural tourism development. The coordination of the two necessitates first planning and then the benign interaction of the two under its supervision. After a lot of thorough investigation and research, the rural tourism products are positioned as folk custom experience tours, and the folk culture of the whole country is transferred and copied to Yunshe Tujia village with good traffic conditions, deep folk culture, and beautiful natural scenery, according to the tourism pattern of “travelling on the mountain, playing at the foot of the mountain, and buying in the city” of Jiangkou tourism. It is jointly developed and invested in by the government, departments, village committees, and villagers. Tourists can directly taste agricultural products or participate in agricultural production activities, gain relevant agricultural production knowledge and have fun, and experience farmers' production labour and rural folk customs. We should improve rural tourism practitioners' and community residents' training. Rural residents have developed a loose, free, and unrestrained habit in their long-term production and life, which is incompatible with the demands of tourism services. Farmers struggle to maintain a mental balance between self-management agricultural production and service reception. The local society's strong regional departmentalism and non-standard characteristics of the concept of hometown, combined with the long history and rich connotation of folk culture, make it mysterious and simple, which is a great draw for tourists. Many resources, such as aboveground and underground resources, national folk customs, human culture, natural environment, and many government departments in charge of planning, construction, tourism, and so on, are involved in the coordinated development of tourism and new rural areas. We should put the idea of serving farmers from various perspectives into action, improve communication and coordination, integrate our own resources, and work together to promote coordinated and healthy tourism and new rural areas.

The article "Interactive Model of Rural Tourism and New Socialist Countryside Construction Using Deep Learning Technology" was retracted in 2023. Reasons: signs of a paper mill; suspected computer-generated content; unreliable results or conclusions; concerns about the data.

## 4. Experimental Results and Analysis

### 4.1. Experimental Data

Empirically speaking, there are three main parameters that affect the model: the number of hidden factors in factorization machine, the number of convolution kernels in convolution network, and the number of neurons in neural network. So, here, we study the influence of these parameters on the model, and we use MSE as the evaluation standard, and the results are shown in Figure 3.

From the results in Figure 3, we can see that when the number of hidden factors reaches 220, the MSE of the model reaches the lowest, on exceeding 220, the performance of the model is basically not improved. When the number of convolution kernels reaches 160, the MSE of the model reaches the lowest, on exceeding 160, the performance of the model is basically not improved. So here, we set the number of hidden factors and convolution kernels to 220 and 160, respectively.

We use different hidden layer schemes to analyze the convolution network which deals with other information in the model, and the results are shown in Table 1.

From Table 1, we can see that increasing the depth and width of the hidden layer can improve the effect, but to a certain extent, the effect will not increase significantly and the amount of calculation will become larger and larger. Therefore, after comprehensive consideration, the two-layer combination of 500 ReLU + 50 ReLU is finally selected as the configuration of the DNN network.

According to the evaluation indicators proposed in the table, the rural tourism and the construction of a new socialist countryside are studied. In this section, the machine learning algorithm is used, and the data mining algorithm is compared with the convolution neural network algorithm proposed in this paper for MSE and MAE. The experimental results are shown in Figures 4 and 5.

From Figures 4–5, it can be seen that the convolution neural network algorithm proposed in this paper has the best performance. Because MSE and MAE reflect the error of prediction score, the lower the value, the higher the recommended accuracy. When the number reaches 80, the MSE value of machine learning algorithm is 2.456, the MSE value of data mining algorithm is 2.324, and the MSE value of convolution neural network algorithm in this paper is 2.102, Therefore, it can be seen from the figure that the MSE value and MAE value of the convolution neural network algorithm proposed in this paper are the lowest among the three methods. In MAE, the same experimental results are obtained. The convolution neural network algorithm is better than the other two algorithms. Although the effect of PMF is better than that of MF, compared with the convolution neural network algorithm proposed in this paper, these two methods do not achieve ideal performance, mainly because these two methods cannot use other information except scoring information.

The article "Interactive Model of Rural Tourism and New Socialist Countryside Construction Using Deep Learning Technology" was retracted in 2023. Reasons: signs of a paper mill; suspected computer-generated content; unreliable results or conclusions; concerns about the data.

### 4.2. Influence of Parameter Setting on Model

In this experiment, we generate prediction scores for the user travel service items in the test set and analyze their errors through MSE. Machine learning algorithm, data mining algorithm, and convolution neural network algorithm are used to analyze the personalization generated for each user according to the prediction score. Precision criteria reflects accuracy and sensitivity, as shown in Figure 6.

It can be seen from Figure 6 that the sensitivity and accuracy of the convolution neural network algorithm proposed in this paper are the first among the three algorithms. Compared with other algorithms, CNN algorithm can make good use of some basic information and comment text information, and also make use of the hidden interaction between these information, which other algorithms do not have. Therefore, their accuracy and sensitivity are lower than those of convolution neural network algorithm.

In order to evaluate the performance and response delay of this model, this paper randomly selects three interface URLs for testing and takes the average response time and the average amount of transmitted data as the final test results. The performance test results are shown in Table 2.

It can be seen from the average value in Table 2 that the average response time and the average amount of data transmitted are within an acceptable and reasonable range. That is, the system can meet the normal use of users.

Under the optimal experimental configuration, the length of word embedding vector is 130, the average number of multiple points at the coding end multiplied by the number of attention layers is 1, and the convergence curve of CNN model on tourinterest data set is shown in Figure 7.

It can be seen from Figure 7 that the value of RMSE is lower when the CNN model uses position coding at the coding end of tourinterest data set. This shows that location coding can make full use of the semantic location information between words in the user's comment information, so as to learn the user's potential interest characteristics and obtain high model prediction performance. From the graph, it can be concluded that the model is convergent.

The article "Interactive Model of Rural Tourism and New Socialist Countryside Construction Using Deep Learning Technology" was retracted in 2023. Reasons: signs of a paper mill; suspected computer-generated content; unreliable results or conclusions; concerns about the data.

The deep learning technology is applied to simulate and predict the suitability of high-grade tourist attractions. The convolution neural network algorithm in the deep learning network is an abstract representation of the shallow neurons. The deep neurons learnt more abstract features of the impact factors, and mine the hidden information between the spatial pattern of the scenic spot and its impact factors. Compared with the traditional neural network algorithm, the simulation results are more reliable. As a large-scale traffic line, the railway line cannot go deep into the scenic spot. Tourists can choose other lines to replace it. Therefore, the law between the railway line and high-level scenic spots is not obvious, as shown in Table 3.

As can be seen from Table 3, the areas that are extremely suitable for developing high-grade tourist attractions are mature and developed in terms of natural environment and social development, which are characterized by high altitude, large vegetation coverage, close distance to provincial capitals and prefecture-level cities, and close distance to national, provincial, and county roads. In this way, the combination of rural tourism with the extension of agricultural industrial chain and agricultural industrialization can not only improve the rural industrial structure and promote the sustainable and healthy development of agricultural economy, but also increase diversified rural tourism resources and promote the construction of new socialist countryside.

## 5. Conclusions

In the face of traditional rural culture, Chinese urban culture presents another cultural form. In the process of development, Chinese urban culture has been impacted by Western culture, which has penetrated the factors of Western culture. It is a hybrid of Chinese and Western culture, and it is difficult to preserve the most original cultural face of China itself. This paper only discusses the relationship between new rural construction and rural tourism development, and the interactive relationship between rural tourism and new rural construction. The convolution neural network algorithm based on deep learning is used to study rural tourism and new socialist rural construction. The convolution neural network algorithm proposed in this paper has the best performance. Since MSE and MAE reflect the error of prediction score, the lower the value, the higher the accuracy of recommendation. When the number reaches 80, the MSE value of machine learning algorithm is 2.456, that of data mining algorithm is 2.324, and that of convolutional neural network algorithm in this paper is 2.102. It can be concluded that the MSE and MAE values of the convolution neural network algorithm proposed in this paper are the lowest of the three methods. Rural tourism should follow the principles of adjusting measures to local conditions, rational distribution and highlighting characteristics, and make an overall plan for regional tourism development. Under the deep learning convolution neural network algorithm, the rural tourism development planning is incorporated into the new rural construction planning, the strategic position of rural tourism in the new rural construction is determined, the rural tourism construction is regarded as an important subsystem of the new rural construction, the sustainable development and characteristic construction of rural tourism, the protection of architectural style and cultural landscape, and the impact of modern architecture on primitive ancient villages and ecological villages are emphasized, emphasize the destruction of ethnic villages and the construction of liveable and tourable villages.

The article "Interactive Model of Rural Tourism and New Socialist Countryside Construction Using Deep Learning Technology" was retracted in 2023. Reasons: signs of a paper mill; suspected computer-generated content; unreliable results or conclusions; concerns about the data.

## Figures and Tables

**Figure 1:** CNN model diagram.

**Figure 2:** Structure diagram of self-encoder.

**Figure 3:** Influence of different methods on prediction results. (a) Number of hidden factors (b) number of convolution kernels.

**Figure 4:** MSE comparison of different algorithms.

**Figure 5:** MAE comparison of different algorithms.

**Figure 6:** Accuracy of different algorithms.

**Figure 7:** Convergence diagram of CNN model.

**Table 1:** Effects of different hidden layers on performance.

Hidden layer	MSE
Without	1.752
25 ReLU	1.702
50 ReLU	1.697
100 ReLU	1.692
50ReLU + 25ReLU	1.681

**Table 2:** Performance test results.

Interface address	Function	Response time	Amount of data
/All_scene/	Return to all attractions	0.35	9.2
/Scene_recommend/	Recommended attractions page	3.56	4.2
/Scene/1553/	Return to the scenic spot with id 1553	0.26	2.2
Average value	—	1.134	4.52

**Table 3:** Statistical results of deep learning simulation of scenic spot pattern.

Suitability zoning	DEM	NDVI	Provincial capital	Prefecture-level city	Provincial highway	Railway
Less suitable area	1.565	0.05	731.58	224.07	58.24	112.53
Moderate and low suitable area	2.251	0.08	569.67	236.83	82.41	146.57
Medium-high suitable area	1.617	0.34	290.73	126.51	31.22	77.52
Extremely suitable area	2.848	0.35	279.09	104.32	27.75	120.94

## Data Availability

The data used to support the findings of this study are available from the corresponding author upon request.
